The article "Evaluation of the Antibacterial Efficacy of QMix and AgNP Solutions in Root Canals of Primary Molars: An In-Vitro Study" was published in 2022. Journal: Cureus.

# Evaluation of the Antibacterial Efficacy of QMix and AgNP Solutions in Root Canals of Primary Molars: An In-Vitro Study

**DOI:** 10.7759/cureus.28877

**Published:** 2022-09-07

**Authors:** Dania Alkhourbotly, Mohamed K Altinawi, Rouaida Abou-Samra, Hasan M Alzoubi, Abedulrahman K Ebrahim

**Affiliations:** 1 Department of Pediatric Dentistry, Damascus University, Damascus, SYR; 2 Department of Pedodontics and Preventive Dentistry, Damascus University, Damascus, SYR; 3 Department of Chemistry and Biochemistry, Damascus University, Damascus, SYR; 4 Department of Endodontics, Damascus University, Damascus, SYR

**Keywords:** primary molars, enterococcus faecalis, antibacterial efficacy, sodium hypochlorite, qmix, irrigation

## Abstract

Purpose

The study aimed to evaluate QMix^2in1^ and silver nanoparticles (AgNPs) solution in eliminating *Enterococcus faecalis* (*E*. *faecalis*) bacteria within root canals of primary molars.

Materials and methods

The study sample consisted of 45 extracted primary molars, which were divided into three groups: Group 1 (control) NaOCl 5.25%, Group 2 (experimental) QMix^2 in 1^, and Group 3 (experimental) AgNPs 4000 ppm. The root canals were sterilized within an autoclave and then contaminated with *E*. *faecalis* bacteria. The root canals were irrigated for five minutes in a quantity of 3 ml using a 31-gauge irrigation needle, and then bacterial smears were taken.

Results

Sodium hypochlorite, AgNPs, and QMix^2in1^ effectively reduced the bacterial count of Enterococcus within root canals of primary molars. There were statistical differences between all groups. QMix^2in1^ solution showed the greatest antibacterial efficacy, then NaOCl solution and AgNPs solution.

Conclusion

All irrigation solutions used are effective in eliminating *E*. *faecalis*. QMix^2in1^ can be considered a good alternative to sodium hypochlorite in irrigation root canals of primary teeth.

## Introduction

Primary teeth play the role of a space maintainer that directs the eruption of permanent teeth to their optimal position in the dental arch. Therefore, preserving primary teeth in the dental arch free from pathological injuries is extremely important [1].

The treatment often includes root canals when primary teeth are infected with dental caries. Therefore, the successful outcome of pulpectomy depends on the disinfection of the root canal system, which aims to eliminate or reduce microscopic microorganisms and their toxic products from root canals [2].

Endodontic treatment of primary teeth presents a real challenge due to anatomical complications such as accessory and abnormal canals [3]. In addition, exposure to dentinal tubules as a result of physiological resorption can lead to structural alterations and increased root surface permeability to various bacterial toxins [4]. Moreover, internal resorption can further modify the root canal system [4].

The article "Evaluation of the Antibacterial Efficacy of QMix and AgNP Solutions in Root Canals of Primary Molars: An In-Vitro Study" was published in 2022. Journal: Cureus.

The necrotic pulp and periapical lesions contain a large number of polymorphic bacteria [5]. *Enterococcus faecalis (E. faecalis)* bacteria has been mentioned with increasing frequency as a serious challenge in endodontic therapy because it is the most common post-endodontic infection. In addition, it is most resistant to environmental conditions (*E. faecalis* can survive in extremely hard environments with high pH levels, temperatures range from 10 to 45°C, and can survive at 60°C for 30 minutes) and many types of dressing materials [6].

Evidence has shown that necrotic tissues, microorganisms, and their products remain within the dentinal tubules and areas of internal resorption, which cause periapical inflammation. Thus, chemo-mechanical debridement is essential by using a clinically effective irrigant that can also aid in removing organic residues [2].

Sodium hypochlorite's tissue dissolution and antimicrobial properties make it one of the most widely recommended irrigants when used in concentrations between 0.5% and 5.25%. However, the serious damage caused by its exit to the apical area, even in small amounts, puts a question mark on its high abrasive ability. This may lead to damage of permanent tooth buds due to potential absorption areas in pediatric patients [2].

QMix^2in1^ consists of a mixture of ethylenediamine tetraacetic acid (EDTA) 17%, chlorhexidine 2%, and surfactants. This mixture can remove the smear layer efficiently, has a strong antibacterial effect, and has good biocompatibility with minimal cytotoxicity. Moreover, the effect of QMix^2in1^ on the color and micro-hardness of dentin is low [7]. Rapid developments in nanotechnology have led to a significant increase in the use of nanoparticles, especially silver nanoparticles (AgNPs), in various fields, including dentistry [8]. Due to the small particle size (usually 1 to 100 nm) and large surface area, the antibacterial properties of AgNPs greatly outperform the molecular shape of silver [9]. Therefore, this study aimed to compare the antibacterial efficacy of sodium hypochlorite, QMix^2in1^, and AgNPs as irrigants against *E. faecalis* in the primary root canal.

## Materials and methods

Study sample

A comparative in vitro study to evaluate the antibacterial activity of NaOCl 5.25%, AgNPs 4000 ppm, and QMix^2in1^ against *E. faecalis*. The study protocol was approved by the Scientific Research and Postgraduate Board of Damascus University, Ethics Committee of Damascus University, Damascus, Syria (IRB No. UDDS-453-23082019/SRC-1450). The sample size was determined using a sample size calculation program (PS: Power and Sample Size Calculation version 3.0.43). Sample size calculation produced a required sample size of 15 primary teeth per group to detect a significant difference (90% power, two-sided 5% significance level). The study sample consisted of 45 extracted primary molars that were divided randomly using http://www.randomization.com into three groups (n=15) according to irrigant used: Group 1 (control) NaOCl 5.25%, Group 2 (experimental) QMix^2in1^, and Group 3 (experimental) AgNPs 4000 ppm. A uni-blinded was also adopted in this study so that the examiner would not know about the applied irrigant. The exclusion criteria were: root resorption of more than a third of the root, teeth that have had previous endodontic treatment, calcified canals, and the presence of fractures or cracks.

The article "Evaluation of the Antibacterial Efficacy of QMix and AgNP Solutions in Root Canals of Primary Molars: An In-Vitro Study" was published in 2022. Journal: Cureus.

Teeth samples preparation

After tooth extraction, the root surface was cleaned using ultrasonic to remove ligaments and tissue remnants, the crowns were cut with diamond discs, root canals were prepared using K-file f with saline, and then the samples were immersed in saline. Rotary preparation was done with Kedo-S files where the D1 Kedo-S rotary file was used (Reeganz Dental Care Pvt Ltd). Then the roots were dried. Phosphorous acid 37% was applied, followed by washing, drying, bonding for 20 seconds, and then applying composite to seal the apical foramen. Next, the roots were coated with two layers of nail polish to prevent bacterial infiltration. Then a cotton ball was placed in the orifices of each root, then sealed with a temporary restoration. Next, the roots were placed in acryl models using a previously prepared rubber model. After the hardening of acryl was completed, the temporary restoration and cotton ball were removed, and the samples were entered into autoclaved at 121°C for 15 minutes. After sterilization, three samples were taken randomly from the total sample, and bacterial smears were taken from them to ensure the samples' sterility and that they were cultured negative.

Sample contamination

*E. faecalis* was isolated from canals infected with an abscess in the Department of Pediatric Dentistry, Damascus University, and then cultured until the appropriate concentration was reached. A special differential test called the bile esculin test (selective test for *E. faecalis*) was used. The sample was incubated with *E. faecalis* in brain heart infusion (BHI) at 37°C. A 30-gauge needle was used to inject the suspension into the root canal. Then, the teeth were incubated at 37°C and left for 48 hours to allow bacterial growth.

The article "Evaluation of the Antibacterial Efficacy of QMix and AgNP Solutions in Root Canals of Primary Molars: An In-Vitro Study" was published in 2022. Journal: Cureus.

Initial enumeration of bacterial colony units

After the incubation period, the primary bacterial smear was taken from each of the canals as follows: the canal was filled with saline, and a circumferential preparation was performed with H-file. The smear was taken using a paper point compatible with the measurement of the final preparation file, and it was left for 10 seconds and then transferred to a sterile Eppendorf containing 1 ml of saline. The smear was repeated three times to obtain an accurate bacterial count. Then the tube containing the paper points was shaken for 1 minute with a Biovortex device to ensure homogeneity of the solution. Three dilutions were performed to determine the appropriate countable dilution as follows:

Dilution 0

A 50 μm of the solution in the Eppendorf tube was taken by a micropipette and cultured on a pre-equipped sectioned Petri dish.

Dilution 1

A 10:1 dilution was performed to change the volume from 1.0 mL to 10 mL by adding 1.0 bacterial suspension to 9.0 mL of serum in a sterile glass tube. A total of 50 μm of the solution in the diluted glass tube was taken and cultured in a sectioned Petri dish.

Dilution 2

A 100:1 dilution was performed by adding 1.0 ml of the 10:1 solution to 9.0 ml of serum in a sterile glass tube, thus reducing the suspension concentration by a factor of 100 ml. A total of 50 µm of the solution was taken from the diluted 100:1 glass tube and cultured in the same Petri dish.

After 48 hours, the dishes were taken out of the incubator, and the microbial units were counted using a colony counting device. Then, these bacterial units were converted into logarithm numbers to facilitate statistical analysis. These extensions were performed to know the bacterial counts of each canal before applying the irrigation protocol to them where dilution No. 2 has been approved.

Irrigation protocol

The root canals were irrigated for five minutes in a quantity of 3 ml using a 31-gauge NaviTip (Ultradent Products Inc, South Jordan, UT) irrigation needle. Next, they were washed with 10 ml of saline to remove traces of the irrigant solution. Next, the canal was filled with saline, and a circumferential preparation was performed with H-file. The smear was then taken using a paper point compatible with the measurement of the final preparation file, and it was left for 10 seconds and then transferred to a sterile Eppendorf containing 1 ml of saline. The smear was repeated three times to obtain an accurate bacterial count. Then the tube containing the paper points was shaken for one minute with a Biovortex device to ensure homogeneity of the solution and cultured on a bile esculin Petri dish (Figures 1-3).

The article "Evaluation of the Antibacterial Efficacy of QMix and AgNP Solutions in Root Canals of Primary Molars: An In-Vitro Study" was published in 2022. Journal: Cureus.

**Figure 1:** Sample of AgNPs group (A) before irrigation, (B) after irrigation. AgNPs: Silver nanoparticles.

**Figure 2:** Sample of sodium hypochlorite group (A) before irrigation, (B) after irrigation.

**Figure 3:** Sample of QMix group (A) before irrigation, (B) after irrigation.

Statistical analysis was performed using the SPSS 21.0 software (IBM, Armonk, NY, USA). The data were analyzed with one-way ANOVA and Kruskal-Wallis tests. The testing was performed at α=0.05 (P<0.05).

## Results

The sample consisted of 45 palatal root canals of primary upper second molars and distal root canals of primary lower second molars, divided into three equal main groups (33.33%) according to irrigant used (NaOCl 5.25%, QMix^2in1^, and AgNPs 4000 ppm). In addition, descriptive statistics were conducted for the decimal logarithm of the number of bacteria, which included the arithmetic mean, SD, median, and maximum and minimum values ​​for each group before and after irrigation, as shown in Table 1.

**Table 1:** Basic sample characteristics. AgNPs: Silver nanoparticles.

Studied stage	Irrigant used	Arithmetic mean	SD	Maximum values	Minimum values
Before Irrigation	NaOCl	7.95	0.184	8.179	7.639
	QMix^2in1^	7.963	0.179	8.166	7.653
	AgNPs	7.939	0.176	8.166	7.627
After Irrigation	NaOCl	0.872	0.856	2.000	0.000
	QMix^2in1^	0.000	0.000	0.000	0.000
	AgNPs	1.988	1.109	3.158	0.000

One-way ANOVA test was conducted to study the significance of the differences in the mean decimal logarithm of the number of bacteria between study groups before irrigation (P-value = 0.937), and the Kruskal-Wallis test to study the significance of the differences after irrigation (P-value = 0.000), as shown in Table 2.

**Table 2:** One-way ANOVA and Kruskal-Wallis tests results.

Studied variable	Studied stage	Chi value or F	P-value	Significance of the differences
The decimal logarithm of the number of bacteria	Before irrigation	0.65^F^	0.937	No statistical differences
	After irrigation	23.02	0.000	Statistical differences

To find out which of the groups is statistically different from the other, a pairwise comparison was made using the Mann-Whitney U test, as shown in Table 3. Again, there were statistical differences between all groups. Returning to the table of arithmetic averages of the irrigant groups after irrigation, we note that the mean decimal logarithm of the number of bacteria is lowest in the QMix group, then the NaOCl group, and the AgNPs group.

**Table 3:** Mann-Whitney U test result. AgNPs: Silver nanoparticles.

Studied stage	Irrigant (1)	Irrigant (2)	Z-value	P-value	Significance of the differences
After irrigation	NaOCl	QMix^2in1^	3.209-	0.001	Statistical differences
		AgNPs	3.098-	0.002	Statistical differences
	QMix^2in1^	AgNPs	-4.215	0.000	Statistical differences

The article "Evaluation of the Antibacterial Efficacy of QMix and AgNP Solutions in Root Canals of Primary Molars: An In-Vitro Study" was published in 2022. Journal: Cureus.

## Discussion

Currently, sodium hypochlorite is the best irrigant solution for root canals, as it is considered the most widely used and common in dentistry. It has antibacterial activity by releasing hypochlorous acid (HOCL), which in turn performs an oxidative action on the sulfhydryl groups of bacterial enzymes, which disrupts the metabolism processes of bacteria [10]. However, it is toxic when extruded to periapical tissues and can damage permanent tooth buds. In addition to its unpleasant taste and odor, direct application of sodium hypochlorite can be harmful as it is associated with the cellular destruction of tissues [11]. Because of the many limitations of sodium hypochlorite solution and to reach the ideal irrigant in root canal treatment, the efficacy of alternative irrigants for endodontic treatments (QMix^2in1^ and AgNPs) has been investigated.

QMix^2in1^ was developed in collaboration with Dr. Markus Haapasalo, Head of the Department of Endodontics at the University of British Columbia. QMix^2in1^ is a ready-to-use liquid requiring no mixing and is effective in removing the smear layer and bacteria such as *E. faecalis* with a single application [12]. QMix is ​​a mixture of antimicrobial agents (CHX 2%), calcium chelating agent PAM (EDTA 17%), saline, and surfactant [13]. QMix also showed durability of up to 120 days because it contains chlorhexidine, and it penetrates dentin canals with a depth of up to 500 microns without causing erosion to the dentin [14]. AgNPs can adhere to and penetrate the cell walls of both Gram-positive and Gram-negative bacteria, disrupting cell function by releasing silver ions; thus, they are used to treat and prevent drug-resistant microorganisms and inhibit biofilm formation [15]. Silver ions interact with three main components of a bacteria cell to produce a bactericidal effect: peptidoglycan layer and plasma membrane, DNA, and bacterial proteins [16]. *E. faecalis* is a selective Gram-positive anaerobe that causes opportunistic infections. It is most closely associated with endodontic failures and periapical tissue inflammation [17]. *E. faecalis* has been used in several previous studies that examined the efficacy of irrigant and dressing materials within root canals [18]. The apical foramen of teeth was closed with composite to transform the inner canal space into a closed system to simulate clinical conditions, and this is what was adopted in this research as a root canal in the presence of the surrounding tissues tends to be a closed-ended system [19]. The irrigant protocol was standardized in terms of time and volume, as the irrigant time, according to previous studies, ranged between 30 seconds and 10 minutes, while the irrigant volume, according to previous studies, ranged between 0.05 ml and 15 ml. The canals in this study were irrigated for five minutes with an amount of 3 ml of irrigant [20]. Bacterial smears were accomplished using sterile paper points, but before taking the bacterial smears, a sterile H-file was used that has an inlet and outlet movement along the root canal, thus obtaining a more realistic bacterial smear [21].

The article "Evaluation of the Antibacterial Efficacy of QMix and AgNP Solutions in Root Canals of Primary Molars: An In-Vitro Study" was published in 2022. Journal: Cureus.

The results of this study showed that all irrigation solutions were effective bacterial count in primary root canals. However, QMix^2in1^ solution showed the most significant antibacterial efficacy, then NaOCl solution and AgNPs solution.

The superiority of the QMix solution was attributed to its materials that have antibacterial properties and the ability to remove the smear layer at the same time [5]. The addition of surfactants to QMix^2in1^ improved the wettability of this solution and thus improved its ability to penetrate further into the root canal. The potential benefit of bisbiguanide in this mixture was its ability to prevent microbial colonization on the surface of the dentin. However, the calcium chelating agent could damage the wall of Gram-negative bacterial cells by removing (Mg+2 and Ca+2) from the bacterial cell membrane and increasing its permeability [22].

The results of this study confirmed what was found by Kishore RS and Saurav S that QMix had a stronger effect on *E. faecalis* bacteria than sodium hypochlorite and that sodium hypochlorite needed to stay inside the root canal for a long time to affect the bacteria within the abnormalities of canals [23]. Furthermore, this study also agreed with Elakanti S et al. and Bindu S et al. that QMix was superior to sodium hypochlorite solution in its antibacterial action against *E. faecalis* [22,24].

The results of this study differed from both Ordinola-Zapata R et al. and Ye WH et al., where sodium hypochlorite outperformed QMix in its antibacterial activity [25,26]. The reason may be that irrigation time to QMix was not enough to allow it to be better distributed within the canal. However, an irrigation time of five minutes seems more reasonable than the 60-90 seconds recommended by the manufacturer. A study by Ma J et al. showed that QMix is ​​as effective as 6% sodium hypochlorite against *E. faecalis*, confirming the results of this study [27]. This study agrees with Kangarlou A et al. study, which evaluated the antibacterial activity of each sodium hypochlorite solution at different concentrations (1.125%, 2.5%, 5.25%) with different concentrations of AgNPs solution (25 ppm, 50 ppm, 100 ppm, 200 ppm, 400 ppm, 4000 ppm) where the greatest antibacterial activity belonged to sodium hypochlorite groups (2.5%, 5.25%) and the silver particle solution had acceptable activity and its antibacterial properties were improved by increasing the concentration of Ag+ [28]. It also agreed with Moradi F et al. study, where all teeth treated with nanoparticles showed a positive reduction in bacterial growth [29]. While the current study differed from Purushotham M et al. study, which showed that the effectiveness of a solution of AgNPs is higher than the effectiveness of 2.5% sodium hypochlorite solution and 2% chlorhexidine solution in reducing the number of bacterial units of *E. faecalis* bacteria. This difference may be attributed to the fact that Purushotham M et al. study used ethanol and hydroxide sodium as a solvent that can reduce the surface tension of the AgNP solution and may help increase the penetration of the solution into dentinal cannulas and may have a role in enhancing its antibacterial activity, while in this study distilled water was the solvent for AgNPs [30]. The present study does not use a negative control group, and this is the major limitation of the present study. In addition, the present study does not evaluate different mL of the irrigating solution.

The article "Evaluation of the Antibacterial Efficacy of QMix and AgNP Solutions in Root Canals of Primary Molars: An In-Vitro Study" was published in 2022. Journal: Cureus.

## Conclusions

The effectiveness of the QMix^2in1^ solution is higher than that of each of the 5.52% sodium hypochlorite and AgNPs (4000 ppm) solutions in reducing the number of bacterial units of *E. faecalis*. The effectiveness of the 5.52% sodium hypochlorite solution was higher than the AgNPs (4000 ppm) solution in reducing the number of bacterial units of *E. faecalis*. Therefore, the solution of AgNPs (4000 ppm) was the least effective.
